# Exposure to Ambient Air Pollutant PM_10_ in the Second Trimester of Pregnancy Is Associated with Preterm Birth: A Birth-Based Health Information Cohort Study

This article has been retracted.

**DOI:** 10.1155/2022/1008538

**Published:** 2022-06-22

**Authors:** Pengying Xiao, Lijun Wang, Yingjie Yao, Yu Chang, Jianghou Hou

**Affiliations:** Clinical Research Center of Kunming Maternal and Child Health Hospital, Kunming 650031, China

## Abstract

**Objectives:**

We evaluated the effects of exposure to high concentrations of particulate matter (PM)_10_ on preterm birth (PTB) and identified a critical concentration of PM_10_ that could lead to PTB *via* a birth-based health information cohort study.

**Methods:**

We conducted a birth-based cohort study consisting of nonanomalous singleton births at 22-42 weeks. PTB was defined as babies born alive before 37 weeks of pregnancy. Pregnancy period exposure averages were estimated for PM_10_ based on the China National Environmental Monitoring Centre (CNEMC). Pregnant women who lived within 50 km of the monitor station were recruited into this study. Logistic regression analyses were performed to determine the association between PTB and exposure to PM_10_ at different pregnancy periods with adjustment for confounding factors.

**Results:**

The relative frequency of PTB was 8.7% in the study cohort of 5,291 singleton live births. A total of 1137 women had a high level of PM_10_ exposure (≥60 *μ*g/m^3^) in the second trimester of pregnancy. The average concentrations of PM_10_ in the first, second, and third trimesters of pregnancy and throughout pregnancy were 53.8 *μ*g/m^3^, 54.2 *μ*g/m^3^, 55.6 *μ*g/m^3^, and 54.3 *μ*g/m^3^, respectively. The generalized additive model (GAM) analysis showed that there was a nonlinear correlation between PM_10_ and PTB in the second trimester of pregnancy (*P* < 0.001). The adjusted odds ratio between PTB and low concentration PM_10_ exposure (PM_10_ < 60 *μ*g/m^3^) in the second trimester of pregnancy was 1.01 (95% CI 0.95-1.05). However, high PM_10_ exposure (PM_10_ ≥ 60 *μ*g/m^3^) in the second trimester of pregnancy had an increased PTB risk even after adjustment for coexisting risk factors with an adjusted odds ratio of 1.78 (95% CI 1.69-1.87), and the incidence of PTB increased with an increase in PM_10_ exposure.

**Conclusions:**

Our research discovered that exposure to high levels of PM_10_ increases the risk of PTB and the second trimester is the most vulnerable gestational period to ambient air pollution exposure. PM_10_ concentrations more than 60 *μ*g/m^3^ are detrimental to pregnant women in their second trimester. This study has implications for health informatics-oriented healthcare decision support systems.

## 1. Introduction

The primary cause of newborn illness and death is preterm birth (PTB) [1]. PTB is expected to occur at a rate ranging from 5% to 13% in industrialized nations [2]. Additionally, PTB has been shown to increase life-long morbidities, such as cardiovascular disease, diabetes, and some types of cancer [3]. Although several risk factors, such as maternal age, alcohol use, smoking, hypertension, diabetes, and infection during pregnancy, are thought to be related to the risk of preterm delivery [4], these variables may not account for all causes of PTB. Numerous studies have shown that environmental variables, such as air pollution, may play a significant role in the risk of PTB.

Environmental pollutants have an increasingly significant impact on human health, especially ambient particulate matter (PM) pollution. Ambient PM pollution has become one of the most important public health risks. The term “ambient PM pollution” refers to a diverse array of airborne particles ranging in size from a few hundredths of a micrometer to visible particles as large as 100 m. Prolonged exposure to ambient PM may result in heart and lung illnesses. The majority of research has been on PM with aerodynamic dimensions less than 10 m (PM_10_) or less than 2.5 m (PM_2.5_), which may impair placental development, disrupt normal gestational processes, and cause PTB [5].

Some studies have reported on the association between PTB and elevated ambient PM levels [6–9]. However, the threshold of PM_10_ level on PTB risk has not been confirmed. China, as a developing country, has a serious problem of environmental PM pollution with the continuous industrial and social development. In 2021, the average PM_10_ concentration in China is 54 *μ*g/m^3^. It is necessary to investigate the relationship between environmental PM pollution and PTB in the country. Clinical studies have found that ultrasonic measurement of the cervical length, measurements of amniotic fluid cytokine and chemokine levels, and sense of coherence 13-item version (SOC-13) scale score in the second trimester of pregnancy can effectively screen women with an increased risk of PTB, which indicates that the second trimester of pregnancy is a sensitive period closely related to the occurrence of PTB [10–12]. Therefore, our study has focused on the second trimester of pregnancy to investigate the correlation between PM_10_ and PTB.

Given the discrepancy between ambient PM pollution and PTB risk and the scarcity of research on high PM_10_ levels, it is critical to explain the link between PM_10_ exposure and PTB risk in China by performing large-scale population studies. We performed a birth cohort research in Kunming, China, adjusting for significant confounders, to examine the connection between PM_10_ and the risk of PTB and to establish a risk threshold for PM_10_ concentration exposure.

## 2. Methods

### 2.1. Participant Profiles

A birth cohort research was performed on births occurring between January 1, 2016, and December 31, 2017, utilizing the Kunming Maternal and Child Health Hospital's database. Pregnant women who presented to the hospital for delivery of singleton newborns between 22 and 42 weeks of gestation without any significant congenital defects, who were not suffering from a mental disorder, and who were 18 years or older were eligible for this study. The Medical Ethics Committee of Kunming Maternal and Child Health Hospital in China authorized all research protocols. To prevent fixed cohort bias, the study population included all babies conceived between January 1, 2016, and December 31, 2017. The study period began 22 weeks before the start of the research and ended 42 weeks before the conclusion of the study.

The estimated date of conception and resultant gestational age (in days) were calculated using the first day of the mother's last menstrual cycle. The primary exclusion criteria were multiple gestation pregnancies, the absence of critical information (e.g., parity, delivery date, and last menstrual cycle), gestational age of less than 22 weeks or more than 42 weeks, numerous, repeated maternal visits, and any congenital abnormalities (Figure 1). After eliminating women who fulfilled the exclusion criteria, a total of 11,514 pregnancies that satisfied the inclusion criteria were originally recruited, and 5,291 pregnancies were included in the analyses.

### 2.2. Exposure Assessment

Data of PM_10_ concentrations were obtained from the China National Environmental Monitoring Centre (CNEMC) (http://www.cnemc.cn/). The home and work addresses of participants were within 50 kilometers of the nearest monitoring sites. The 24-hour average PM_10_ concentration was measured for the period from January 2016 to December 2017 in Kunming by CNEMC. The daily exposure to PM_10_ was adjusted according to the monitoring week to obtain the annual average of PM_10_ at the monitoring site. The exposure window was defined as the period of the second trimester (14-26 weeks) [13].

### 2.3. Preterm Birth

PTB was defined as less than 37 completed weeks of gestational age [14]. The gestational age was determined using the starting day of the previous menstrual cycle (LMP). During early pregnancy follow-up visits, obstetricians noted women's LMP time (no later than 12 weeks after conception). Each woman was questioned again about the time of LMP at the postpartum follow-up appointment (no later than six weeks following birth), and gestational age was computed using these two records. PTB was classified according to the gestational age as moderate or late PTB (32–37 completed weeks), very PTB (28–32 completed weeks), and extremely PTB (28 completed weeks) [15].

### 2.4. Covariates

Variables or potential confounding effects that had biological importance for PTB were included as adjustments [16, 17]. We adjusted for maternal age, parity (0, 1, 2, ≥3), preeclampsia (yes/no), history of cesarean section (yes/no), maternal anemia (yes/no), maternal obesity (yes/no), and diabetes (yes/no) from the baseline data of the birth cohort. Conception season (spring: March-May; summer: June-August; fall: September-November; winter: December-February) and maternal smoking during pregnancy (yes/no) were included from the early gestation follow-up data. We also adjusted for the mode of delivery (vaginal delivery/Cesarean section) and baby's sex (male/female) from the postpartum follow-up data. The year of conception was also adjusted to eliminate the long-term effects of pollution levels on birth outcomes.

### 2.5. Statistical Analysis

To characterize the demographic, medical, pregnancy outcome, and PM_10_ concentration features, descriptive statistics were used. The association between trimester-specific and total pregnancy PM_10_ exposure and PTB was estimated using a generalized additive model (GAM), adjusting for confounding factors, such as maternal age, parity, preeclampsia, season of conception, history of cesarean section, maternal anemia, maternal obesity, and diabetes. We further used a two-stage linear regression model to capture the potential nonlinear effect of PM_10_ concentration on PTB and explored the turning point of PM_10_ concentration that had a significant positive correlation with PTB through an “exploratory” analysis. We additionally performed stratified analyses of variables, and interaction terms with PM_10_ concentration (<60 or ≥60 *μ*g/m^3^) were used to evaluate whether the effect modifications were statistically significant or not.

Furthermore, we utilized a sensitivity analysis in the main model to check the robustness of the estimated associations. Univariate analysis was performed to evaluate the variables considered possible moderators of PTB, and the statistically significant confounding factors were identified to be adjustment factors. Analyses were performed using the statistical packages R and EmpowerStats (R). Results were reported as the odds ratios (OR) and 95% confidence intervals (CI) for the association between PM_10_ exposure during pregnancy and risk of PTB. *P* values < 0.05 were considered statistically significant.

## 3. Results

The study population included 5,291 singleton live births: 462 (8.7%) were preterm and 4,829 were term births. Among the PTBs, 409 were moderate or late PTBs and 53 were very PTBs (VPTBs) or extremely PTBs (ExPTBs). The mean concentrations of PM_10_ exposure over the first, second, and third trimesters of pregnancy and the entire pregnancy were 53.8 *μ*g/m^3^, 54.2 *μ*g/m^3^, 55.6 *μ*g/m^3^, and 54.3 *μ*g/m^3^, respectively. Furthermore, of the 5291 infants included in our study, 1137 had a high level of PM_10_ (≥60 *μ*g/m^3^) in the second trimester of pregnancy (Table 1). Univariate analysis was performed to identify factors associated with PTB. Factors with significant associations included parity, year and season of conception, cesarean, and preeclampsia (Table S1).

In order to explore the relationship between PM_10_ exposure during pregnancy and gestational age or PTB, a GAM was used (Figure 2). With adjustment for season of conception, parity, maternal age, preeclampsia, history of cesarean section, maternal anemia, maternal obesity, and diabetes, a nonlinear association was found between PM_10_ exposure and gestational age (*P* < 0.001), and consistent associations were found between PM_10_ exposure and PTB (*P* < 0.001) in the second trimester of pregnancy. When we examined the relationships according to the PM_10_ exposure level, we discovered that exposure to a higher PM_10_ concentration (≥60 *μ*g/m^3^) during the second trimester of pregnancy was clearly associated with an elevated risk of PTB.

Table 2 presents the crude and adjusted OR (with 95% CI) of gestational age or PTB associated with PM_10_ exposure in the second trimester of pregnancy. In the crude analysis, we observed a consistent relationship between PM_10_ exposure (<60 *μ*g/m^3^ or ≥60 *μ*g/m^3^) and gestational age. Exposure to high PM_10_levels ≥ 60 *μ*g/m^3^ in the second trimester of pregnancy was significantly associated with an increased risk of PTB, with an OR of 1.71 (95% CI: 1.63, 1.78). However, no significant association between exposure to PM_10_levels < 60 *μ*g/m^3^ in the second trimester of pregnancy and PTB was observed, with an OR of 1.02 (95% CI: 1.00, 1.04). In the adjusted models, similar association was found between gestational age and PM_10_ exposure. We also found that exposure to high PM_10_levels ≥ 60 *μ*g/m^3^ in the second trimester of pregnancy was still significantly associated with an increased risk of PTB, with an OR of 1.78 (95% CI: 1.69, 1.87), and we found that the risk of PTB was increased by 78% for each 1 *μ*g/m^3^ increase in PM_10_ exposure in the second trimester of pregnancy. There was no significant association between exposure to PM_10_levels < 60 *μ*g/m^3^ in the second trimester of pregnancy and PTB, with an OR of 1.01 (95% CI: 0.95, 1.05).

Furthermore, we conducted a stratified analysis by grouping confounding variables, such as season of conception, parity, maternal age, preeclampsia, history of cesarean section, maternal anemia, maternal obesity, and diabetes. After excluding the confounding variables, exposure to high PM_10_ levels (≥60 *μ*g/m^3^) in the second trimester of pregnancy was significantly associated with an increased risk of PTB, but there was no significant correlation between exposure to PM_10_ levels (<60 *μ*g/m^3^) in the second trimester of pregnancy and PTB. The results indicated the robustness of the association between exposure to high PM_10_ levels and PTB (Table 3).

## 4. Discussion

Preterm birth is a significant public health issue. It is not only the biggest cause of newborn death [18], but it also has significant long-term consequences, including asthma, metabolic abnormalities, and disability [19]. Our investigation established a link between PM in the air and unfavorable birth outcomes. Exposure to high levels (PM_10_ ≥ 60 *μ*g/m^3^) during the second trimester of pregnancy was substantially related with an elevated risk of PTB in our research population. On the other hand, exposure to PM_10_ < 60 *μ*g/m^3^ levels during the second trimester of pregnancy was not related to an increased risk of PTB. As a result, we determined that a PM_10_ level of 60 *μ*g/m^3^ considerably increased the risk of PTB. Additionally, we discovered similar correlations between PM_10_ exposure and PTB across a variety of possible confounding populations.

Previous studies have reported various results for the relationship between ambient PM_10_ and risk of PTB. A prospective birth cohort study in Wuhan in China reported an about 2% increase (OR = 1.02; 95% CI: 1.02, 1.03) in PTB per 5 *μ*g/m^3^ increase in PM_10_ during pregnancy [20]. A study performed in Australia observed a 15% (OR = 1.15; 95% CI: 1.06, 1.25) elevated risk for PTB per 4.5 *μ*g/m^3^ increase in PM_10_ during the first trimester [21]. A study performed in Uruguay reported a 10% (OR = 1.10; 95% CI: 1.03, 1.19) increase in PTB per 10 *μ*g/m^3^ increase in PM_10_ during the third trimester [22]. A Korean study observed a 7% (OR = 1.07; 95% CI: 1.01, 1.14) increase in PTB per 16.53 *μ*g/m^3^ increase in PM_10_ during the first or third trimester [23]. These studies reported that PM_10_ exposure during pregnancy was associated with PTB, with ORs ranging from 1.01 to 1.15, which was confirmed in our study. In addition, we found a non-linear relationship between PM_10_ exposure and risk of PTB during pregnancy, and the actual risk of PTB with an adjustment OR of 1.78 (95% CI: 1.69-1.87, *P* < 0.001) was observed for PM_10_ ≥ 60 *μ*g/m^3^.

The threshold for the PM_10_ level that causes adverse birth outcomes is not clearly defined. Pregnant women in our study lived in areas with a high PM_10_ pollution level (>50 *μ*g/m^3^), which is much higher than the limit value stated by WHO (PM_10_ < 40 *μ*g/m^3^). Using the exposure response curve, we found that the threshold for the PM_10_ level was 60 *μ*g/m^3^. In addition, we identified a significant association between PM_10_ exposure above the threshold and PTB risk. However, when PM_10_ exposure was below the threshold, no increase in the risk for PTB was identified. Therefore, it is recommended that the PM_10_ level should remain below 60 *μ*g/m^3^, which may be safe for PTB risk.

Although many studies have reported about the relation between the risk of PTB and exposure to the PM10 sensitivity window during pregnancy, the conclusions are still controversial. Some studies have suggested that exposure to high levels of PM_10_ during the first and/or third trimester of pregnancy had a greater impact on PTB than exposure over the second trimester [24]. However, other reports have observed the effect of PM_10_ exposure during the second trimester of pregnancy on PTB was more significant [25]. In our study, we found a significant correlation between PTB and PM_10_ exposure in the second trimester of pregnancy.

The biological mechanism of PTB caused by airborne PM is still unclear. Some studies have found that immune cells in maternal and umbilical cord blood of pregnant women exposed to PM_10_ presented the characteristics of inflammation [26]. Particulate matter may affect the overall health of pregnant women by inducing airway inflammation and oxidative stress. Cytokines and peroxides produced in the course of immune inflammation may also have adverse effects on fetal growth [27]. It can be assumed that systemic oxidative stress and inflammatory response may be one of the mechanisms underlying the risk of PTB in pregnant women exposed to PM [28]. To further explore these research findings, additional research is needed so as to expand the research areas and population cohorts.

Our study also had several limitations. First, the limited number of monitors (seven monitors in this study) in the population study area might have affected the accuracy of exposure estimation. Although more than 90% of women lived within 50 km of a monitor, exposure misclassification was still possible for residents living far away from monitors. However, this type of misclassification should exist equally among the research groups. Second, air pollution exposure was estimated using data from government monitors in most epidemiology studies, but these data might be inconsistent with the actual level of personal exposure due to the difference in the indoor/outdoor activity environment. However, such exposure assessment errors might generally underestimate the risk of PTB associated with air pollution [29]. Finally, the study population was recruited from only one Chinese city, which weakened the generalizability of the results to other cities or other countries. However, because of the limitations in obtaining hospital data, we have currently completed 2 years of data analysis. We will continue to collect 5 or 10 years of data for analysis in the future.

In conclusion, our study suggests that women exposed to high level of PM_10_ (≥60 *μ*g/m^3^) over the course of pregnancy are at an increased risk for PTB. The risks of different exposure time windows are consistent. This study defines a safe threshold for PM_10_ exposure, which supports policy-makers to design air pollution policies in China.

## Figures and Tables

**Figure 1:** Flow diagram of the study population.

**Figure 2:** Associations between air pollutant PM_10_ and risk of PTB or gestational age in the second trimester of pregnancy. (a) A nonlinear association between PM_10_ exposure during the second trimester and gestational age was found (*P* < 0.001) in a generalized additive model (GAM). (b) Consistent association between PM_10_ exposure during the second trimester and PTB was found (*P* < 0.001) in a GAM model. The solid red line represents the smooth curve fit between variables. The blue bands represent the 95% of confidence interval from the fit. All adjusted for season of conception, parity, maternal age, preeclampsia, history of cesarean section, maternal anemia, maternal obesity, and diabetes.

**Table 1:** Maternal and fetal characteristics in the birth cohort.

Characteristic	Data
Maternal	
Age, mean ± SD	29.8 ± 4.6
Gestational age (wk), mean ± SD	38.8 ± 1.7
Parity, no. (%)	
1	2857 (54.3)
2	2250 (42.8)
≥3	150 (2.9)
Year of conception, no. (%)	
2015	1686 (31.9)
2016	3605 (68.1)
Season of conception, no. (%)	
Spring	1265 (23.9)
Summer	1043 (19.7)
Autumn	1613 (30.5)
Winter	1370 (25.9)
Mode of delivery, no. (%)	
Vaginal	5063 (95.7)
Cesarean	228 (4.3)
Preeclampsia, no. (%)	173 (3.3)
Diabetes, no. (%)	642 (12.1)
Maternal obesity, no. (%)	140 (2.6)
Maternal anemia, no. (%)	2147 (40.6)
History of cesarean section, no. (%)	1009 (19.1)
Infant	
Birth weight (g), mean ± SD	3009.7 ± 366.4
Sex of infant, no. (%)	
Male	2495 (47.1)
Female	2296 (43.4)
Missing	500(9.5)
Term birth, no. (%)	4829 (91.3%)
PTB, no. (%)	462 (8.7)
Moderate or later preterm ≥ 224, <259	409 (7.7)
VPTB	52 (1.0)
ExPTB	1 (0)
Mean concentration of PM_10_ (*μ*g/m^3^), mean ± SD	
First trimester	53.8 ± 7.9
Second trimester	54.2 ± 9.6
Third trimester	55.6 ± 11.1
Entire pregnancy	54.3 ± 3.7
PM_10_ exposure during the second trimester (%)	
<60 *μ*g/m^3^	4154 (78.5)
≥60 *μ*g/m^3^	1137 (21.5)

PM_10_: particulate matter with aerodynamic diameters ≤ 10 *μ*m; PTB: preterm birth; VPTB: very preterm birth; ExPTB: extremely preterm birth. Dichotomous variables are presented as percent of total for each characteristic.

**Table 2:** Crude and adjusted odd ratios for the risk of gestational age (wk) and PTB caused by PM_10_ exposure in the second trimester of pregnancy.

Outcome	Crude		Model I		Model II	
	OR/*β* (95% CI)	*P* value	OR/*β* (95% CI)	*P* value	OR/*β* (95% CI)	*P* value
Gestational age (wk)						
PM_10_ < 60 (*μ*g/m^3^)	0.02 (0.01, 0.02)	<0.001	0.02 (0.01, 0.03)	<0.001	0.02 (0.01, 0.03)	<0.001
PM_10_ ≥ 60 (*μ*g/m^3^)	-0.47 (-0.48, -0.46)	<0.001	-0.48 (-0.50, -0.47)	<0.001	-0.48 (-0.49, -0.47)	<0.001
PTB						
PM_10_ < 60*(μg*/m^3^)	1.02 (1.00, 1.04)	0.129	1.00 (0.95, 1.06)	0.883	1.01 (0.95, 1.05)	0.992
PM_10_ ≥ 60 (*μ*g/m^3^)	1.71 (1.63, 1.78)	<0.001	1.75 (1.67, 1.83)	<0.001	1.78 (1.69, 1.87)	<0.001

OR: odds ratio; CI: confidence interval. Model I adjusted for season of conception and maternal age. Model II adjusted for season of conception, parity, maternal age, preeclampsia, history of cesarean section, maternal anemia, maternal obesity, and diabetes.

**Table 3:** Logistic regression of factors associated with PTB in the second trimester of pregnancy.

Subgroup	PM_10_ < 60 (*μ*g/m^3^)		PM_10_ ≥ 60 (*μ*g/m^3^)	
	OR (95% CI)	*P* value	OR (95% CI)	*P* value
Maternal age				
<25	1.02 (0.82, 1.28)	0.852	1.88 (1.61, 2.19)	<0.001
25-29	1.03 (0.94, 1.13)	0.574	1.75 (1.62, 1.88)	<0.001
30-34	0.99 (0.90, 1.07)	0.733	1.77 (1.61, 1.95)	<0.001
≥35	0.97 (0.87, 1.09)	0.628	1.86 (1.61, 2.14)	<0.001
Sex of infant				
Male	0.97 (0.90, 1.05)	0.485	1.87 (1.71, 2.03)	<0.001
Female	1.01 (0.93, 1.09)	0.868	1.72 (1.61, 1.85)	<0.001
Missing	1.19 (0.85, 1.67)	0.315	1.81 (1.49, 2.19)	<0.001
Parity				
1	0.99 (0.92, 1.07)	0.847	1.78 (1.66, 1.91)	<0.001
2	1.02 (0.94, 1.11)	0.589	1.78 (1.65, 1.93)	<0.001
≥3	0.85 (0.67, 1.07)	0.173	1.90 (1.39, 2.59)	<0.001
Preeclampsia				
No	0.99 (0.94, 1.05)	0.850	1.79 (1.70, 1.89)	<0.001
Yes	1.48 (0.62, 3.52)	0.379	1.61 (1.38, 1.88)	<0.001
Diabetes				
No	1.01 (0.96, 1.08)	0.648	1.81 (1.71, 1.92)	<0.001
Yes	0.95 (0.85, 1.06)	0.359	1.63 (1.45, 1.83)	<0.001
Maternal obesity				
No	1.00 (0.95, 1.05)	0.9464	1.76 (1.68, 1.85)	<0.001
Yes	—		—	
Maternal anemia				
No	1.00 (0.93, 1.07)	0.964	1.72 (1.62, 1.83)	<0.001
Yes	1.00 (0.92, 1.08)	0.956	1.87 (1.72, 2.04)	<0.001
Mode of delivery				
Vaginal	0.97 (0.40, 2.36)	0.941	—	
Cesarean	1.03 (0.96, 1.11)	0.397	1.80 (1.69, 1.91)	<0.001
History of cesarean section				
No	0.99 (0.94, 1.05)	0.805	1.81 (1.71, 1.92)	<0.001
Yes	1.03 (0.91, 1.16)	0.627	1.67 (1.51, 1.85)	<0.001
Year of conception				
2015	1.07 (0.80, 1.43)	0.6656	—	
2016	1.04 (0.99, 1.09)	0.0909	8.04 (6.15, 10.52)	<0.001
Season of conception				
Spring	0.93 (0.81, 1.07)	0.2986	2.57 (1.95, 3.40)	<0.001
Summer	1.06 (0.90, 1.24)	0.5187	—	
Autumn	1.01 (0.92, 1.11)	0.8591	1.24 (0.73, 2.09)	0.4271
Winter	2.01 (1.28, 3.15)	0.0023	1.59 (1.50, 1.68)	<0.001

Odds ratio estimates for covariates are adjusted for other factors listed in the first column of the table as well as season of conception, parity, maternal age, preeclampsia, history of cesarean section, maternal anemia, maternal obesity, and diabetes. The odds ratio estimates for PM_10_exposure < 60 *μ*g/m^3^ or ≥60 *μ*g/m^3^ are from separate models with adjustment for the same covariates as listed above.

## Data Availability

No data were used to support this study.

## Supplementary Materials

Supplementary Materials Table S1: univariate analysis of factors associated with PTB.
